The article "Pharmacokinetic Difference of Six Active Constituents of Huangqi Liuyi Decoction between Control and Diabetic Nephropathy Mouse Models" was published in 2022. Journal: Int J Anal Chem.

# Pharmacokinetic Difference of Six Active Constituents of Huangqi Liuyi Decoction between Control and Diabetic Nephropathy Mouse Models

**DOI:** 10.1155/2022/7602992

**Published:** 2022-05-25

**Authors:** Qun Wang, Ya Shi, Xingde Liu, Ting Liu, Yongjun Li, Xinli Song, Xiaolan Chen, Yang Jin, Wen Liu, Yonglin Wang, Zipeng Gong

**Affiliations:** ^1^Guizhou University of Traditional Chinese Medicine, Huaxi University Town, Guiyang 550025, China; ^2^Guizhou Provincial Key Laboratory of Pharmaceutics, Guizhou Medical University, Beijing Road, Guiyang 550000, China

## Abstract

Huangqi Liuyi decoction is a famous traditional Chinese medicine (TCM) that has been widely used in China for the management of diabetes since the Song Dynasty. Today, it is commonly used for treating diabetic nephropathy (DN). Our previous experimental studies have suggested that the mixture HQD, containing astragalus saponin, astragalus flavone, astragalus polysaccharide, and glycyrrhetinic acid, could be used for the treatment of DN and to improve renal function. The objective of this study was to develop a sensitive and reliable high-performance liquid chromatography-tandem mass spectrometry method for simultaneous quantitation of astragaloside IV, calycosin-7-O-*β*-D-glucoside, calycosin-glucuronide, ononin, formononetin, and glycyrrhizic acid, which are the main active constituents in HQD, and to compare the pharmacokinetics of these active constituents in control and DN mice orally treated with HQD. The results indicated that the pharmacokinetic parameters of HQD were significantly different between the control and DN mouse groups. The absorption of HQD in the DN mice was greater than that in control mice.

## 1. Introduction

Diabetic nephropathy (DN), one of the most serious complications of diabetes mellitus, is an irreversible, progressive disease characterized by a continuous decline in the glomerular filtration rate, proteinuria, microalbuminuria, and increased blood pressure [1–3], with most cases eventually progressing to end-stage renal disease [4]. Prevention of or early treatment for DN may improve the survival rate and quality of life for patients, which would help to avoid the extremely high costs of renal treatment for end-stage renal disease as well as for other complications [5]. Traditional Chinese medicines (TCMs) have been widely applied in the clinical treatment of various diseases for a long time [6]. In particular, TCMs offer unique advantages in the prevention of diabetic complications because of limited side effects and/or less toxicity [7, 8]. Huangqi Liuyi decoction (HQD) is a popular TCM formula that has been used in China since the Song Dynasty. It is composed of *Radix Astragali* and *Radix Glycyrrhizae*. Research has shown that HQD can significantly decrease the fasting blood glucose and improve the degree of pathological damage to the kidneys in DN rats [9, 10]. In preliminary pharmacodynamic research work of our research group, the results confirmed that the main active components of HQD for the treatment of DN are astragalus saponin, astragalus flavone, astragalus polysaccharide, and glycyrrhizic acid, and the mixture of these four active components (HQD) can significantly delay the pathogenesis of DN in db/db mice. Moreover, the difference in pharmacodynamics was not statistically significant between HQD and Huangqi Liuyi decoction.

The article "Pharmacokinetic Difference of Six Active Constituents of Huangqi Liuyi Decoction between Control and Diabetic Nephropathy Mouse Models" was published in 2022. Journal: Int J Anal Chem.

In recent years, an increasing amount of research has shown that the pharmacokinetic parameter of traditional Chinese medicine can be affected by the disease states [11]. Nevertheless, the major recipients of these drugs are patients. In a pathological state, the severity of the pathological state can have significant effects on the absorption, distribution, metabolism, and excretion of the drug, which is undeviatingly associated with the efficiency and side effects of the drug. The pharmacokinetic study of TCM under physiological and pathological conditions will support the rational application of TCMs in the clinic. Concerning the clinically safe medication of renal diseases, pharmacokinetic research about TCM can contribute more credible information, which helps significantly to elucidate the safety and effectiveness of drugs during the treatment process [12–14].

Previous reports have focused on the pharmacological effects of HQD while also encompassing some pharmacokinetic investigation. However, most pharmacokinetic studies of effective constituents of HQD to date have conducted their investigations under normal conditions. Based on the above reason, in this study, a high-performance liquid chromatography-tandem mass spectrometry (HPLC-MS/MS) method for the simultaneous determination of six active ingredients of HQD, including astragaloside IV, calycosin-7-O-*β*-D-glucoside, calycosin-glucuronide, ononin, formononetin, and glycyrrhizic acid in mouse plasma, was first established. Then, the pharmacokinetic differences of these six active ingredients were investigated between control and DN miceafter the oral administration of HQD, which would provide some reference for the dose adjustment of HQD in clinic.

## 2. Materials and Methods

### 2.1. Materials

The reference standards of astragaloside IV (purity >99.0%), calycosin-7-O-*β*-D-glucoside (purity >98.0%), calycosin-glucuronide (purity >98.0%), formononetin (purity >98.0%), ononin (purity >98.0%), glycyrrhetinic acid (purity >99.0%), puerarin (internal standard, IS, purity >98.0%), and digoxin (IS, purity >98.0%) were obtained from the National Institute for the Control of Pharmaceutical and Biological Products (Beijing, China). Acetonitrile and methanol (HPLC grade) were purchased from Merck KGaA (Darmstadt, Germany). Other chemicals used were of reagent grade or analytical grade.

The article "Pharmacokinetic Difference of Six Active Constituents of Huangqi Liuyi Decoction between Control and Diabetic Nephropathy Mouse Models" was published in 2022. Journal: Int J Anal Chem.

A mixture of four active constituents from HQD was produced. The composition is as follows: astragalus saponin with a 72.04% content, which was 2.69% astragaloside IV; astragalus flavone with a 69.43% content, which was 1.62% calycosin-7-O-*β*-D-glucoside, 1.42% calycosin-glucuronide, 0.89% ononin, and 0.31% formononetin; glycyrrhetinic acid with a 72.04% content; and astragalus polysaccharides with a 65.82% content.

### 2.2. Animals

Ten-week-old db/db mice (weighing 45 ± 5 g) and db/m mice (weighing 20 ± 2 g) were obtained from the Model Animal Research Center of Nanjing University (Qualified number SCXK(Su)2018-0008) and raised in the specific-pathogen-free (SPF) laboratory of the Experimental Animal Center of Guizhou Medical University for two weeks. Ten-week-old db/db mice can develop nephropathy at 12 weeks of age. All mice were housed in polypropylene cages and maintained under standard conditions (25°C ± 20°C; relative humidity, 60% ± 5%; and light-dark cycle of 12 h each). The protocols for all of the animal studies were approved by the Animal Ethics Committee of Guizhou Medical University (NO1702080).

### 2.3. Conditions of HPLC-MS/MS

Figure 1 shows the chemical structure of six analytes. An Acquity HPLC system (Shimadzu Corp., Kyoto, Japan) equipped with a Q-Trap® 5500 triple quadruple mass spectrometer (AB Sciex, Framingham, MA, USA) was employed for HPLC-MS/MS. The chromatographic conditions of the four constituents of HQD were achieved on an Excel2C18-AR system (100 × 2.1 mm, 2 *μ*m; Advanced Chromatography Technologies Ltd., Aberdeen, UK) maintained at 30°C. Analysis was completed with a gradient elution of 0.1% formic acid (*A*) and acetonitrile (*B*) and a flow rate of 0.4 mL/min. The gradient elution was as follows: 0 to 0.6 min (90% A), 0.6 to 2 min (90 ⟶ 70% *A*), 2 to 6 min (70 ⟶ 35% *A*), 6 to 8 min (35 ⟶ 10% *A*), 8 to 9 min (10 ⟶ 10% *A*), 9 to 9.1 min (10 ⟶ 90% *A*), and 9.1 to 12 min (90% *A*). For MS/MS detection, an electrospray ionization in a multireaction monitoring mode was operated with polarity switching between negative and positive ion modes. The mass spectrometer parameters were set as follows: ion spray voltage at 5.5 kV (+) and −4.5 kV (−), source temperature at 600°C, nebulizer pressure at 55 psi, curtain gasat 30 psi, and auxiliary gas at 55 psi. The multiple reaction monitoring (MRM) analysis was conducted by monitoring theprecursor ion to produce ion transitions of *m/z* 807.4 ⟶ 627.4 for astragaloside IV, 447.1 ⟶ 285.2 for calycosin-7-O-*β*-D-glucoside, 285.3 ⟶ 213.2 for calycosin-glucuronide, 267.0 ⟶ 252.0 for formononetin, 431.3 ⟶ 269.1 for ononin, 824.4 ⟶ 309.4 for glycyrrhizic acid, 417.1 ⟶ 267.1 for puerarin, and 825.3 ⟶ 649.5 for digoxin.  Figure 2 shows the mass spectra of six analytes.

The article "Pharmacokinetic Difference of Six Active Constituents of Huangqi Liuyi Decoction between Control and Diabetic Nephropathy Mouse Models" was published in 2022. Journal: Int J Anal Chem.

### 2.4. Plasma Sample Preparation

The whole blood samples were centrifuged at 4°C for 10 min at 3,000 rpm. A 50 *μ*L aliquot of the supernatant was placed in the sample tubes and combined with 25 *μ*L of methanoic acid (1 M), 25 *μ*L of methanol, and 10 *μ*L of internal standard solution (0.75 µg/mL of puerarin and 6.02 µg/mL of digoxin). Then, the mixture was added to 200 *μ*L of methanol to be de-proteinated. Subsequently, the tubes were vortex-mixed for 5 min at 60 Hz and centrifuged for 10 min at 12,000 rpm. An aliquot of the upper organic layers was transferred to sample tubes and evaporated to dryness with a nitrogen-blowing instrument (Organomation, Berlin, MA, USA) at 40°C. The residue was sonicated with 50 *μ*L of 50% methanol and then centrifuged for 10 min at 10,000 rpm. Then, 1 *μ*L of supernatant was injected into the HPLC-MS/MS system for analysis.

### 2.5. Preparation of Standard Samples

Stock solutions were separately prepared by dissolving astragaloside IV (5.34 mg), calycosin-7-O-*β*-D-glucoside (5.05 mg), calycosin-glucuronide (5.19 mg), ononin (5.07 mg), formononetin (5.23 mg), and glycyrrhizic acid (5.09 mg) into methanol to yield the following concentrations: astragaloside IV (0.534 mg/mL), calycosin-7-O-*β*-D-glucoside (0.505 mg/mL), calycosin-glucuronide (0.519 mg/mL), ononin (0.507 mg/mL), formononetin (0.523 mg/mL), and glycyrrhizic acid (0.509 mg/mL). A series of working standard solutions were prepared by dilution of the stock solution with methanol. All the stock and working solutions were stored at 4°C and brought to room temperature before use. Quality control samples representing the low, medium, and high concentrations were separately prepared for each analyte.

### 2.6. Method Validation

#### 2.6.1. Specificity

The blank plasma sample chromatogram was conducted under the method of plasma sample preparation using 50 *μ*L of blank plasma taken from each mouse, except for adding IS. The blank plasma was spiked with astragaloside IV, calycosin-7-O-*β*-D-glucoside, calycosin-glucuronide, ononin, formononetin, and glycyrrhizic acid, and IS chromatogram, and plasma samples obtained after the oral administration of HQD were treated in the same fashion.

The article "Pharmacokinetic Difference of Six Active Constituents of Huangqi Liuyi Decoction between Control and Diabetic Nephropathy Mouse Models" was published in 2022. Journal: Int J Anal Chem.

#### 2.6.2. Calibration Curves and Linearity

The stock solution of astragaloside IV, calycosin-7-O-*β*-D-glucoside, calycosin-glucuronide, ononin, formononetin, and glycyrrhizic acid was closely weighed and added to methanol as desired for dilution to create a series of mixed working solutions. Calibration standards were prepared by spiking the appropriate standard working solutions with 50 *μ*L of blank plasma to yield calibration concentrations of six analytes. The calibration curves were fitted using a weighted least‐squares linearity regression. The calibration curves were obtained by plotting the peak area ratio compared with the concentration of the six analytes with linear regression using standard plasma samples at seven concentrations.

#### 2.6.3. Accuracy and Precision

The quality control samples at three concentration levels of six kinds of analytes of mouse plasma were prepared and operated in parallel according to the above methods of plasma sample preparation, with each concentration analyzed by six replicates. Assay precision was calculated by using the relative standard deviation (RSD, %) and variance. Accuracy was expressed as mean ± standard deviation.

#### 2.6.4. Extraction Efficiency and Matrix Effect

Blank plasma solutions (50 *μ*L) spiked with the quality control sample at three concentration levels (low, medium, and high), each with six replicates, were prepared according to the above methods of plasma sample preparation and regarded as sample *A*. Another 50 *μ*L of blank plasma was prepared according to the above methods of plasma sample preparation, and sample *B* was obtained by mixing standard solution and IS into the obtained supernatant followed by evaporation. Then, the residue was reconstituted with 50 *μ*L of methanol. Sample *C* was acquired by mixing standard solution and IS followed by evaporation. Then, the residue was reconstituted with 50 *μ*L of methanol. Extraction efficiency was calculated by the peak area ratio (*A*/*B*), and the matrix effect was calculated by the peak area ratio (*B*/*C*).

#### 2.6.5. Stability

Quality control samples at three concentrations of three kinds of constituents of mouse plasma were prepared to investigate the stability of six analytes of processed plasma samples After storing them at room temperature (approximately 25°C) for 24 hours, we froze them (−20°C) for 48 hours, and repeated freezing and thawing three times. They were then processed based on the abovementioned plasma sample processing method and measured by HPLC-MS/MS.

### 2.7. Pharmacokinetic Analysis

The model and control mice were randomly divided into two groups. All mice were fasted overnight (12 h) prior to a single oral administration of HQD (1.64 g/kg), and 0.2 mL of blood was collected from the heart of each animal at 0, 10, and 30 min and 1, 1.5, 2, 3, 4, 6, 8, 12, 24, and 48 h. The blood concentration at each time point was the average value from eight mice. The pharmacokinetic parameters of six ingredients were calculated by WinNoLin version 6.4 using a noncompartment model. All of the data are presented as mean ± standard deviation values. Statistical analysis between the two groups was performed using SPSS version 23 (IBM Corporation, Armonk, NY, USA). *P* ≤ 0.01 and *P* ≤ 0.05 between the two groups were statistically different.

The article "Pharmacokinetic Difference of Six Active Constituents of Huangqi Liuyi Decoction between Control and Diabetic Nephropathy Mouse Models" was published in 2022. Journal: Int J Anal Chem.

## 3. Results and Discussion

### 3.1. Evaluation of the Animal Model

Table 1 shows that the biochemical indicators of blood glucose, serum creatinine, blood urea nitrogen, and 24-hour urinary albumin were significantly increased (*P* < 0.05) in 12-week-old db/db mice. As compared to control mice, the kidneys of 12-week-old db/db mice were obviously enlarged and their surface was not smooth. Renal pathological sectioning revealed an obvious degree of collagen fiber (blue part) in the renal tubules and glomerular basement membrane of 12-week-old db/db mice. We concluded that diabetic db/db mice can develop DN at 12 weeks of age. Therefore, the 12-week db/db mice were used as the model group. The kidney shape and pathological sectioning of 12-week db/db and db/m control mice are seen in Figure 3.

The db/db mouse is a mutant-type mouse with a leptin receptor gene defect picked from C57BL/6J mice by the Jackson Laboratory of the United States. It has the features of spontaneously developed type 2 diabetes, and its pathogenesis is very similar to human type 2 diabetes. Db/db mice continuously experience obesity, hyperlipidemia, hyperglycemia, diabetes, and other diabetic symptoms after 4 weeks of age. Then, they began to experience DN after 8–12 weeks [15, 16]. The experimental results showed that the blood glucose, blood creatinine, urea nitrogen, triglycerides, cholesterol, and 24-h urine albumin of 12-week db/db mice were significantly higher than those of the normal control group (*P* < 0.05). The kidney pathological tissue sections of 12-week db/db mice had obvious glomerular and renal tubular lesions. In this case, this experiment used 12-week db/db mice as the DN mouse model, including same-week-old db/m mice as the normal comparison group.

### 3.2. Method Validation

Currently, the commonly applied plasma sample-processing methods principally include solid-phase extraction, liquid-liquid extraction, organic solution protein precipitation, and multiple processing methods [17]. Based on the duality and solubility of saponins and flavonoids examined in this experiment, protein precipitation agents such as methanol, acetonitrile, and ethyl acetate, including the extraction method with *n*-butanol, were examined in the study. The methanol was used as the protein precipitation solvent for the experimental samples. We reviewed 1×, 2×, and 4× methanol as the protein precipitant. When 4× methanol was used as the protein precipitant, the separation of the ingredients was good. Furthermore, the recovery rate could meet the analysis requirements of biological samples. Meanwhile, combining an appropriate amount of formic acid when precipitating proteins with methanol can significantly enhance the recovery rate. The final resolution of the plasma sample-processing method is to acidify the plasma with 1% formic acid solution, then attach methanol to the vortex, and mix for protein precipitation.

The article "Pharmacokinetic Difference of Six Active Constituents of Huangqi Liuyi Decoction between Control and Diabetic Nephropathy Mouse Models" was published in 2022. Journal: Int J Anal Chem.

There are various types of TCMs, with numerous components and complex structures, including a low oral bioavailability. The triple quadrupole mass spectrometer has the advantages of a short analysis time, accurate quantification, and the capacity to examine many components. Currently, it is the most illustrative quantitative analysis instrument in the area of mass spectrometry, and it has been widely used in the pharmacokinetics of multicomponent TCMs [18, 19]. An HPLC-MS/MS method was established to concurrently determine astragaloside IV, calycosin-7-O-*β*-D-glucoside, calycosin-glucuronide, ononin, formononetin, and glycyrrhizic acid in mouse plasma. Additionally, digoxin was chosen as the internal standard substance identified in the negative ion mode. There is no mutual interference with endogenous substances in plasma, which can have a better correction impact. According to the nature of the mixture, methanol/water is used as the liquid mobile phase and 0.1% formic acid is attached to decrease peak tailing and improve the symmetry of the chromatographic peak. Eventually, the chromatographic column ACEExcel2C18-AR (1100 × 2.1 mm, 2 *μ*m; Advanced Chromatography Technologies Ltd., Aberdeen, Scotland) was used. The column temperature was 30°C, and the volume flow was 0.4 mL/min. Moreover, the mobile phase was *A* (water, 0.1% formic acid aqueous solution) and *B* (acetonitrile) gradient elution as HPLC liquid-phase separation conditions. Methodologically confirmed, the method has high sensitivity, good repeatability, accurate results, and high specificity and meets the requirements of biological sample examination and detection.

#### 3.2.1. Specificity

For the chromatograms of the blank plasma sample, the blank plasma spiked with astragaloside IV (1), calycosin-7-O-*β*-D-glucoside (2), calycosin-glucuronide (3), ononin (4), formononetin (5), and glycyrrhizic acid (6), and IS (puerarin and digoxin), and plasma samples obtained after oral administration of HQD are displayed in Figure 4. The results indicated that good separation was observed among the analytes, and no interference from the endogenous substances interfered with the determination of analyte and IS.

The article "Pharmacokinetic Difference of Six Active Constituents of Huangqi Liuyi Decoction between Control and Diabetic Nephropathy Mouse Models" was published in 2022. Journal: Int J Anal Chem.

#### 3.2.2. Calibration Curves and Linearity

The typical equation of linearity ranges and calibration curves for the six analytes are shown in Table 2. The results show that all the correlation coefficients were >0.99, indicating that the concentrations of the six analytes of astragaloside IV, calycosin-7-O-*β*-D-glucoside, calycosin-glucuronide, ononin, formononetin, and glycyrrhizic acid in mouse plasma correlated well within the linearity ranges.

#### 3.2.3. Accuracy and Precision

The results of the intra- and interday precision and accuracy of six analytes in plasma samples are shown in Table 3. The RSD (%) values of intra- and interday precision for all analytes were ≤15%, and the RSD (%) values of accuracy of six analytes were within the range of 81.22%–106.01%, These data suggest that both the precision and accuracy achieved with this method were accurate and reliable, with good repeatability.

#### 3.2.4. Extraction Efficiency and Matrix Effect

The results of the extraction efficiency and matrix effect are shown in Table 4. The extraction efficiency and matrix effect of six analytes at three different concentrations and IS were found to be 82.04%–112.7%, which indicated that the recoveries of the six analytes were precise, consistent, and reproducible at different concentration levels in various plasma biosamples with no significant plasma matrix interference.

#### 3.2.5. Stability

The results of stability are shown in Table 5. The stability test results indicated that the plasma samples had good stability under the three different conditions with a 10% concentration variation compared with the initial values.

### 3.3. Pharmacokinetics of Six Active Ingredients in HQD

The mean plasma concentration-time profiles (*n* = 8) of six active ingredients (astragaloside IV, calycosin-7-O-*β*-D-glucoside, calycosin-glucuronide, ononin, formononetin, and glycyrrhizic acid) after the oral administration of HQD are shown in Figures 5–10. The pharmacokinetic parameters of the six active ingredients are listed in Tables 6–11. The HPLC-MS/MS method was successfully applied to determine the pharmacokinetics of six active ingredients in the plasma of normal and DN mice after a single oral administration of HQD (1.64 g/kg). Following the oral administration of HQD, the area under the curve of six active ingredients (astragaloside IV, calycosin-7-O-*β*-D-glucoside, calycosin-glucuronide, ononin, formononetin, and glycyrrhizic acid) and the *C*_max_ values of astragaloside IV, ononin, and formononetin in the model group were increased (*P* *<* 0.05), while CL_Z_/*F* had slowed down (*P* *<* 0.05). However, the *T*_1/2_ of astragaloside IV, glycyrrhizic acid, and formononetin, and the MRT of glycyrrhizic acid and the *T*_max_ of astragaloside IV in the model group were postponed (*P* *<* 0.05), while the *V*_*Z*_/*F* of astragaloside IV in the model group was slowed down (*P* *<* 0.05). There was no significant difference in other pharmacokinetic parameters.

The article "Pharmacokinetic Difference of Six Active Constituents of Huangqi Liuyi Decoction between Control and Diabetic Nephropathy Mouse Models" was published in 2022. Journal: Int J Anal Chem.

A sensitive, accurate, and rapid HPLC-MS/MS method was developed and validated for the simultaneous quantification of six ingredients of HQD in mouse plasma. Following the oral administration of HQD, the blood concentration level of ononin was lower than the detection line at 8 h, and the blood concentration level of calycosin-7-O-*β*-D-glucoside was lower than the detection line at 6 h. Glucoside was contained in the structure of flavonoids, which are easily metabolized using bacteria after entering the intestine [20, 21]. Meanwhile, calycosin-7-O-*β*-D-glucoside and formononetin were rapidly metabolized into aglycones due to the actions of bacteria in the intestine, resulting in a shortened retention time of the prototype in the body. The mean plasma concentration-time profiles of six components both appeared to have multiple peaks, which could be explained as a phenomenon in two ways. On the one hand, drugs discharged through bile into the intestine can be reabsorbed through the portal vein into the bloodstream. On the other hand, the drug may be absorbed at multiple sites, and interactions with other medications could also cause its blood concentration level to rise again.

Within the HQD, the pharmacokinetic parameters of astragaloside IV, calycosin-7-O-*β*-D-glucoside, calycosin-glucuronide, ononin, formononetin, and glycyrrhizic acid have meaningful diversity in physiological and pathological conditions. Then, in contrast to normal mice, the absorption of six index components in DN mice significantly increased. Their metabolism and elimination were slowed down, and the retention time in the body was imperceptibly longer. This may be because of a modification in the activity or expression of many drug-metabolizing enzymes and transporters implicated in drug absorption and metabolism in the stage of DN that leads to changes in drug absorption and metabolic processes in the body. The kidneys are important secretion and excretion organs of the body. Apart from drugs eliminated by the liver and gallbladder, most drugs are excreted by the kidneys in their original form or as metabolites. The excretion of drugs is the result of the combined effects of nephron filtration, secretion, and reabsorption [22–24]. Consequently, the impairment of renal function may also be one of the reasons for the slowing down of drug elimination.

The article "Pharmacokinetic Difference of Six Active Constituents of Huangqi Liuyi Decoction between Control and Diabetic Nephropathy Mouse Models" was published in 2022. Journal: Int J Anal Chem.

## 4. Conclusions

We have developed a sensitive and reliable HPLC-MS/MS method for simultaneous quantitation of astragaloside IV, calycosin-7-O-*β*-D-glucoside, calycosin-glucuronide, ononin, formononetin, and glycyrrhizic acid, which are the main active constituents in HQD, and compared the pharmacokinetics of these six active ingredients in control and DN mice orally treated with HQD.

## Figures and Tables

**Figure 1:** The chemical structure of six analytes.

**Figure 2:** The mass spectra of six analytes. (a) Astragaloside IV, (b) calycosin-7-O-*β*-D-glucoside, (c) calycosin-glucuronide, (d) ononin, (e) formononetin, (f) glycyrrhetinic acid, (g) puerarin, and (h) digoxin.

**Figure 3:** Observation of the shape of 12-week db/db and db/m control mice (a), renal pathological sectioning of db/m control mice (b), and renal pathological sectioning of 12-week db/db mice (c) (Masson, ×400).

**Figure 4:** The chromatogram of HPLC-MS/MS. Blank plasma sample (a), blank plasma spiked with six ingredients and IS (b), and plasma samples obtained 30 min after oral HQD treatment (c).

**Figure 5:** Concentration-time profiles of astragaloside IV after HQD administration ($\bar{x}$ ± SD, *n* = 8).

**Figure 6:** Concentration-time profiles of glycyrrhizic acid after HQD administration ($\bar{x}$ ± SD, *n* = 8).

**Figure 7:** Concentration-time profiles of calycosin-7-O-*β*-D-glucoside after HQD administration ($\bar{x}$ ± SD, *n* = 8).

**Figure 8:** Concentration-time profiles of calycosin-glucoside after HQD administration ($\bar{x}$ ± SD, *n* = 8).

**Figure 9:** Concentration-time profiles of ononin after HQD administration ($\bar{x}$ ± SD, *n* = 8).

**Figure 10:** Concentration-time profiles of formononetin after HQD administration ($\bar{x}$ ± SD, *n* = 8).

**Table 1:** The biochemical indicators of control and 12-week db/db mice ($\bar{x}$ ± SD, *n* = 6).

Group	Blood glucose (mmol/L)	Serum creatinine (*μ*mol/L)	Urea nitrogen (mmol/L)	Triglyceride (mmol/L)	Cholesterol (mmol/L)	24 h urinary albumin (mg/day)
Control	6.07 ± 0.88	22.84 ± 5.29	6.07 ± 1.31	0.96 ± 0.19	3.03 ± 0.35	17.34 ± 1.36
db/db	18.05 ± 2.87^*∗∗*^	31.49 ± 5.76^*∗*^	7.78 ± 1.23^*∗*^	1.79 ± 0.27^*∗∗*^	3.87 ± 0.51^*∗∗*^	28.44 ± 3.17^*∗∗*^

ps: vs. control group, ^∗^*P* < 0.05, ^∗∗^*P* < 0.01.

**Table 2:** Calibration curve of six analytes in mouse plasma.

Analyte	Linear regression equation	*r*	Linear range (ng/mL)	LLOQ (ng/mL)	LOD (ng/mL)
Astragaloside IV	*Y* = 0.0025*X* + 0.3926	0.9993	10.68–2670	10.68	0.33
Calycosin-7-O-*β*-D-glucoside	*Y* = 0.0375*X* + 0.9606	0.9995	5.05–505	5.05	0.01
Calycosin-glucuronide	*Y* = 0.0208*X* + 0.4845	0.9995	5.19–2595	5.19	0.03
Formononetin	*Y* = 0.0043*X* + 0.1080	0.9992	2.62–523	2.62	0.03
Ononin	*Y* = 0.0033*X* + 0.1591	0.9990	5.07–1014	5.07	0.07
Glycyrrhizic acid	*Y* = 0.0109*X* + 0.5029	0.9995	5.09–3817	5.09	0.04

The article "Pharmacokinetic Difference of Six Active Constituents of Huangqi Liuyi Decoction between Control and Diabetic Nephropathy Mouse Models" was published in 2022. Journal: Int J Anal Chem.

**Table 3:** Intra- and interday precision and accuracy of six analytes in mouse plasma ($\bar{x}$ ± SD, *n* = 6).

Analyte	Concertation of analyte (ng/mL)	Mean ± SD (ng/mL)	Accuracy (%)	Interday precision RSD (%)	Intraday precision RSD (%)
Astragaloside IV	16.02	15.01 ± 0.66	93.68 ± 6.71	4.42	8.47
	801	813.9 ± 74.06	101.6 ± 1.99	9.10	6.56
	1602	1522 ± 107.33	95.03 ± 7.20	7.05	7.08

Calycosin-7-O-*β*-D-glucoside	15.15	15.59 ± 1.55	102.9 ± 5.23	9.94	8.92
	75.75	67.65 ± 5.51	89.31 ± 7.56	8.14	5.39
	151.5	157.8 ± 5.67	104.2 ± 7.83	3.59	6.70

Calycosin-glucuronide	10.38	8.57 ± 0.48	82.57 ± 1.91	2.31	5.57
	519	492.9 ± 23.56	94.98 ± 9.15	4.78	6.10
	1038	927.5 ± 81.62	89.35 ± 7.03	8.80	5.27

Formononetin	5.23	5.02 ± 0.44	95.97 ± 8.32	8.67	6.41
	261.5	266.6 ± 19.86	101.9 ± 7.59	7.45	7.59
	313.8	307.4 ± 41.02	97.83 ± 10.18	13.35	7.10

Ononin	10.41	9.35 ± 0.77	92.24 ± 5.93	8.22	7.61
	507	445.8 ± 32.63	87.93 ± 5.11	7.32	10.16
	1014	1051 ± 60.94	103.6 ± 6.96	5.80	4.40

Glycyrrhizic acid	12.73	11.89 ± 1.3	93.40 ± 10.24	10.96	3.22
	1273	1046 ± 62.99	82.23 ± 1.34	1.62	5.28
	2545	2525 ± 142.15	99.21 ± 3.96	5.63	4.38

**Table 4:** Extraction recovery and matrix effect of six analytes in mouse plasma ($\bar{x}$ ± SD, *n* = 6).

Analyte	Concertation of analyte (ng/mL)	Extraction recovery (%)	RSD %	Matrix effect (%)	RSD %
Astragaloside IV	16.02	99.78 ± 7.56	7.58	87.11 ± 6.52	7.48
	801	106.1 ± 8.53	8.04	94.20 ± 9.33	9.90
	1602	112.7 ± 6.14	5.44	85.36 ± 3.49	4.08

Calycosin-7-O-*β*-D-glucoside	15.15	91.18 ± 3.46	3.80	83.04 ± 2.79	3.35
	75.75	89.05 ± 9.37	10.52	90.46 ± 4.80	5.31
	151.5	94.7 ± 4.23	4.46	101.9 ± 6.78	6.65

Calycosin-glucuronide	10.38	96.56 ± 8.59	8.89	86.86 ± 4.76	5.48
	519	82.39 ± 1.27	1.54	107.90 ± 10.01	9.27
	1038	110.9 ± 7.38	6.66	91.45 ± 7.41	8.11

Formononetin	5.23	103.1 ± 8.40	8.15	90.86 ± 6.58	7.24
	261.5	88.54 ± 5.65	6.38	93.47 ± 7.60	8.13
	313.8	102.8 ± 9.73	9.47	99.22 ± 7.79	7.85

Ononin	10.41	87.28 ± 6.74	7.73	104.42 ± 10.60	10.15
	507	98.92 ± 11.01	11.13	85.95 ± 3.69	4.29
	1014	86.36 ± 4.19	4.85	103.38 ± 10.49	10.15

Glycyrrhizic acid	12.73	90.03 ± 7.80	8.66	83.77 ± 1.92	2.29
	1272.5	95.35 ± 7.06	7.41	93.47 ± 7.60	8.13
	2545	89.83 ± 4.29	4.78	99.22 ± 7.79	7.85

The article "Pharmacokinetic Difference of Six Active Constituents of Huangqi Liuyi Decoction between Control and Diabetic Nephropathy Mouse Models" was published in 2022. Journal: Int J Anal Chem.

**Table 5:** Stability of six analytes in mouse plasma ($\bar{x}$ ± SD, *n* = 6).

Analyte	Concertation of analyte (ng/mL)	Sampler 4 h		−20°C 48 h		Three freeze-thaw	
		Mean ± SD (ng/mL)	RSD (%)	Mean ± SD (ng/mL)	RSD (%)	Mean ± SD (ng/mL)	RSD (%)
Astragaloside IV	16.02	15.76 ± 1.34	8.52	15.17 ± 1.08	7.10	15.58 ± 1.58	10.14
	801	826.8 ± 49.36	5.97	841.1 ± 54.76	6.51	760.6 ± 50.89	6.69
	1602	1591 ± 113.94	7.16	1538 ± 62.14	4.04	1578 ± 72.92	4.62

Calycosin-7-O-*β*-D-glucoside	15.15	14.53 ± 0.93	6.40	14.72 ± 1.34	9.11	14.05 ± 1.31	9.31
	75.75	77.08 ± 4.93	6.39	82.83 ± 7.14	8.62	78.27 ± 2.88	3.68
	151.5	149.2 ± 10.29	6.90	143.8 ± 7.73	5.38	141.4 ± 9.57	6.77

Calycosin-glucuronide	10.38	9.99 ± 0.67	6.69	9.87 ± 0.34	3.42	9.71 ± 0.46	4.69
	519	523.5 ± 19.84	3.79	557.9 ± 50.32	9.02	532.1 ± 25.91	4.87
	1038	1025 ± 78.08	7.62	1031 ± 45.24	4.39	1051 ± 50.02	4.76

Formononetin	5.23	5.47 ± 0.57	10.89	5.58 ± 0.37	6.65	5.35 ± 0.63	11.73
	261.5	245.4 ± 1162.01	13.92	261.5 ± 23.25	8.89	251.2 ± 27.17	10.82
	313.8	311.6 ± 28.6	9.18	322.7 ± 30.69	9.51	308.7 ± 25.75	8.34

Ononin	10.41	9.67 ± 0.73	7.51	9.9 ± 0.46	4.63	9.79 ± 0.74	7.61
	507	505.7 ± 34.19	6.76	469.0 ± 41.13	8.77	475.6 ± 22.73	4.78
	1014	993.2 ± 66.94	6.74	942.6 ± 51.09	5.42	920.9 ± 40.52	4.40

Glycyrrhizic acid	12.73	11.64 ± 1.28	11.01	12.26 ± 0.77	6.27	11.89 ± 1.3	10.97
	1273	1250 ± 68.62	5.49	1186 ± 83.68	7.06	1185 ± 83.68	7.06
	2545	2472 ± 139.15	5.63	2463 ± 104.69	4.25	2414 ± 74.35	3.08

**Table 6:** The pharmacokinetic parameters of astragaloside IV after HQD administration.

Pharmacokinetic parameter	Unit	Astragaloside IV	
		Control group	Model group
*T*_1/2_	h	9.85 ± 0.82	15.11 ± 1.15^*∗∗*^
*T*_max_	h	1.75 ± 0.29	2.75 ± 0.50^*∗*^
*C*_max_	ng/mL	1248 ± 101.7	1882 ± 429.1^*∗*^
AUC_(0–*t*)_	ng^*∗*^h/mL	7624 ± 235.7	14414 ± 952.1^*∗∗*^
AUC_(0–∞)_	ng^*∗*^h/mL	8012 ± 266.8	15710 ± 895.4^*∗∗*^
*V*_Z_/*F*	mL/kg	191756 ± 1417	15025 ± 1133^*∗∗*^
CL_*Z*_/*F*	mL/h/kg	1351 ± 44.04	690.3 ± 39.31^*∗∗*^
MRT_(0–*t*)_	h	9.95 ± 0.47	10.49 ± 1.13
MRT_(0–∞)_	h	12.44 ± 1.19	15.33 ± 1.60

ps: vs. control group, ^∗^*P* < 0.05, ^∗∗^*P* < 0.01.

**Table 7:** The pharmacokinetic parameters of glycyrrhizic acid after HQD administration ($\bar{x}$ ± SD, *n* = 8).

Pharmacokinetic parameter	Unit	Glycyrrhizic acid	
		Control group	Model group
*T*_1/2_	h	9.87 ± 1.64	17.78 ± 3.55^*∗*^
*T*_max_	h	1.38 ± 0.25	1.63 ± 0.25
*C*_max_	ng/mL	1892 ± 513.8	2661 ± 630.1
AUC_(0–*t*)_	ng^*∗*^h/mL	6962 ± 729.8	12174 ± 1374^*∗∗*^
AUC_(0–∞)_	ng^*∗*^h/mL	7152 ± 725.4	13725 ± 1497^*∗∗*^
*V*_Z_/*F*	mL/kg	180200 ± 40486	169076 ± 38405
CL_*Z*_/*F*	mL/h/kg	12618 ± 1340	6590 ± 787.4^*∗∗*^
MRT_(0–*t*)_	h	9.12 ± 0.96	11.48 ± 1.71
MRT_(0–∞)_	h	10.56 ± 0.45	18.49 ± 4.74^*∗*^

ps: vs. control group, ^∗^*P* < 0.05, ^∗∗^*P* < 0.01.

The article "Pharmacokinetic Difference of Six Active Constituents of Huangqi Liuyi Decoction between Control and Diabetic Nephropathy Mouse Models" was published in 2022. Journal: Int J Anal Chem.

**Table 8:** The pharmacokinetic parameters of calycosin-7-O-*β*-D-glucoside after HQD administration ($\bar{x}$ ± SD, *n* = 8).

Pharmacokinetic parameter	Unit	Calycosin-7-O-*β*-D-glucoside	
		Control group	Model group
*T*_1/2_	h	3.22 **±** 0.88	3.85 **±** 2.21
*T*_max_	h	1.13 **±** 0.25	1.25 **±** 0.29
*C*_max_	ng/mL	117.5 **±** 34.19	161.2 **±** 39.84
AUC_(0–*t*)_	ng^*∗*^h/mL	118.3 **±** 12.90	191.0 **±** 15.68^*∗∗*^
AUC_(0–∞)_	ng^*∗*^h/mL	175.7 **±** 22.75	273.9 **±** 49.48^*∗*^
*V*_Z_/*F*	mL/kg	65898 **±** 12674	48618 **±** 20157
CL_*Z*_/*F*	mL/h/kg	14611 **±** 2106	9473 **±** 1511^*∗*^
MRT_(0–*t*)_	h	1.62 **±** 0.21	1.37 **±** 0.11
MRT_(0–∞)_	h	4.27 **±** 1.44	4.30 **±** 1.90

ps: vs. control group, ^∗^*P* < 0.05, ^∗∗^*P* < 0.01.

**Table 9:** The pharmacokinetic parameters of calycosin-glucuronide after HQD administration ($\bar{x}$ ± SD, *n* = 8).

Pharmacokinetic parameter	Unit	Calycosin-glucoside	
		Control group	Model group
*T*_1/2_	h	13.16 **±** 1.74	15.62 **±** 1.50
*T*_max_	h	0.88 **±** 0.25	1.13 **±** 0.25
*C*_max_	ng/mL	704.6 **±** 152.8	954.8 **±** 194.7
AUC_(0–*t*)_	ng^*∗*^h/mL	1851 **±** 264.6	2701 **±** 211.0^*∗∗*^
AUC_(0–∞)_	ng^*∗*^h/mL	2034 **±** 265.9	2977 **±** 218.1^*∗∗*^
*V*_Z_/*F*	mL/kg	21128 **±** 4333	16877 **±** 1939
CL_*Z*_/*F*	mL/h/kg	1110 **±** 144.3	749.9 **±** 55.07^*∗∗*^
MRT_(0–*t*)_	h	10.15 **±** 0.32	10.47 **±** 0.44
MRT_(0–∞)_	h	15.27 **±** 1.08	15.98 **±** 1.87

ps: vs. control group, ^∗^*P* < 0.05, ^∗∗^*P* < 0.01.

**Table 10:** The pharmacokinetic parameters of ononin after HQD administration ($\bar{x}$ ± SD, *n* = 8).

Pharmacokinetic parameter	Unit	Ononin	
		Control group	Model group
*T*_1/2_	h	1.31 **±** 0.02	1.63 **±** 0.83
*T*_max_	h	1.38 **±** 0.25	1.25 **±** 0.29
*C*_max_	ng/mL	351.6 **±** 63.44	677.4 **±** 157.9^*∗*^
AUC_(0–*t*)_	ng^*∗*^h/mL	576.0 **±** 43.31	817.0 **±** 93.25^*∗∗*^
AUC_(0–∞)_	ng^*∗*^h/mL	596.4 **±** 44.22	865.9 **±** 106.9^*∗∗*^
*V*_Z_/*F*	mL/kg	4434.7 **±** 357.0	3739 **±** 1618
CL_*Z*_/*F*	mL/h/kg	2343 **±** 171.8	1633 **±** 226.9^*∗∗*^
MRT_(0–*t*)_	h	1.80 **±** 0.21	1.67 **±** 0.14
MRT_(0–∞)_	h	2.04 **±** 0.27	2.14 **±** 0.32

ps: vs. control group, ^∗^*P* < 0.05, ^∗∗^*P* < 0.01.

**Table 11:** The pharmacokinetic parameters of formononetin after HQD administration ($\bar{x}$ ± SD, *n* = 8).

Pharmacokinetic parameter	Unit	Formononetin	
		Control group	Model group
*T*_1/2_	h	3.17 ± 0.47	4.71 ± 1.17^*∗*^
*T*_max_	h	0.63 ± 0.25	0.75 ± 0.29
*C*_max_	ng/mL	191.1 ± 69.46	354.9 ± 74.35^*∗*^
AUC_(0–*t*)_	ng^*∗*^h/mL	429.4 ± 24.92	645.03 ± 105.8^*∗∗*^
AUC_(0–∞)_	ng^*∗*^h/mL	460.1 ± 32.3	730.61 ± 88.31^*∗∗*^
*V*_Z_/*F*	mL/kg	4791.9 ± 346.9	4569 ± 1498
CL_*Z*_/*F*	mL/h/kg	1047 ± 76.97	664.3 ± 80.3^*∗∗*^
MRT_(0–*t*)_	h	2.92 ± 0.22	3.04 ± 0.28
MRT_(0–∞)_	h	3.83 ± 0.39	4.96 ± 0.96

ps: vs. control group, ^∗^*P* < 0.05, ^∗∗^*P* < 0.01.

The article "Pharmacokinetic Difference of Six Active Constituents of Huangqi Liuyi Decoction between Control and Diabetic Nephropathy Mouse Models" was published in 2022. Journal: Int J Anal Chem.

## Data Availability

The data used to support the finding of this study are included within the article.

## References

[1] Zhang Z. H., Mao J. R., Chen H. (2017). Removal of uremic retention products by hemodialysis is coupled with indiscriminate loss of vital metabolites. *Clinical Biochemistry*.

[2] Xiao X. Y., Ma B., Dong B. J. (2009). Cellular and humoral immune responses in the early stages of diabetic nephropathy in NOD mice. *Journal of Autoimmunity*.

[3] Kopel J., Pena-Hernandez C., Nugent K. (2019). Evolving spectrum of diabetic nephropathy. *World Journal of Diabetes*.

[4] Chen H., Chen L., Liu D. (2017). Combined clinical phenotype and lipidomic analysis reveals the impact of chronic kidney disease on lipid metabolism. *Journal of Proteome Research*.

[5] Correa-Rotter R., Gonzalez-Michaca L. (2005). Early detection and prevention of diabetic nephropathy: a challenge calling for mandatory action for mexico and the developing world. *Kidney International*.

[6] Peng Y. b., Ren D., Song Y. f. (2020). Effects of a combined fucoidan and traditional Chinese medicine formula on hyperglycaemia and diabetic nephropathy in a type II diabetes mellitus rat model. *International Journal of Biological Macromolecules*.

[7] Shi X., Lu X. G., Zhan L. B. (2011). The effects of the Chinese medicine ZiBu PiYin recipe on the hippocampus in a rat model of diabetes-associated cognitive decline: a proteomic analysis. *Diabetologia*.

[8] Sun G. D., Li C. Y., Cui W. P. (2016). Review of herbal traditional Chinese medicine for the treatment of diabetic nephropathy. *Journal of Diabetes Research*.

[9] Xu Y. L., Zheng Y. J., Li Z. (2017). Effect of Huangqi Liuyi Tang on glucose re-absorption via renal tubular epithelial cells in type 2 diabetes model rats. *Chinese Journal of Experimental Traditional Medical Formulae*.

[10] Wen L. M., Xu Y. L., Li Z. (2018). Study on the effects and mechanism of astragalus Liuyi Decoction on type 2 diabetes mellitus rats. *Journal of Chinese Medicinal Materials*.

[11] Gong Z. P., Chen Y., Zhang R. J., Yang Q., Zhu Xx. (2015). Advances on pharmacokinetics of traditional Chinese medicine under disease states. *China Journal of Chinese Materia Medica*.

[12] Zhu S. Y., Wang X., Zheng Z., Zhao X. E., Bai Y., Liu H. (2020). Synchronous measuring of triptolide changes in rat brain and blood and its application to a comparative pharmacokinetic study in normal and Alzheimer’s disease rats. *Journal of Pharmaceutical and Biomedical Analysis*.

The article "Pharmacokinetic Difference of Six Active Constituents of Huangqi Liuyi Decoction between Control and Diabetic Nephropathy Mouse Models" was published in 2022. Journal: Int J Anal Chem.

[13] Zhang W., Fu Z. T., Xie Y. D., Duan Z. W., Wang Y., Fan R. H. (2020). High resolution UPLC-MS/MS method for simultaneous separation and determination of six flavonoids from *semen cuscutae* extract in rat plasma: application to comparative pharmacokinetic studies in normal and kidney-deficient rats. *Natural Product Research*.

[14] Dai X. X., Su S. L., Cai H. D. (2017). Comparative pharmacokinetics of acteoside from total glycoside extracted from leaves of rehmannia and dihuangye total glycoside capsule in normal and diabetic nephropathy rats. *Biomedical Chromatography*.

[15] Appel G. (2013). Detecting and controlling diabetic nephropathy:what do we know. *Cleveland Clinic Journal of Medicine*.

[16] Ponchiardi C., Mauer M., Najafian B. (2013). Temporal profile of diabetic nephropathy pathologic changes. *Current Diabetes Reports*.

[17] Dong J. C., Zeng L. X., Wang X. (2018). Progress on application of biological sample pretreatment technology in pharmacokinetic research. *Traditional Chinese Drug Research and Clinical Pharmacology*.

[18] Bo H., Zhang R. H., Wang X. H. (2018). The application progress of triple quadrupole mass spectrometry in studies of traditional Chinese medicine. *Journal of Inner Mongolia University for Nationalities*.

[19] Liu X. Y., Chen X. Y., Zhong D. Y. (2017). Matrix effects and countermeasure of liquid chromatography-tandem mass spectrometry in bioanalysis. *Journal of Chinese Mass Spectrometry Society*.

[20] Liu L., Zhao X. L., Di L. Q. (2015). Effects of radix saposhnikoviae on metabolism of calycosin-7-O-*β*-D-glucoside in radix astragali by intestinal flora experiment in vitro. *Journal of Nanjing University of Traditional Chinese Medicine*.

[21] Zhang W., Jiang S., Qian D. W. (2014). The interaction between ononin and human intestinal bacteria. *Acta Pharmaceutica Sinica*.

[22] Wang L. N., Lin X., Shen L. (2015). Effect of common clinical diseases on pharmacokinetics of traditional Chinese medicine. *Chinese Journal of Experimental Traditional Medical Formulae*.

[23] Sun G. l., Lin X. (2010). Mechanisms and strategies for targeting drugs to myocardial ischemic regions. *Acta Pharmaceutica Sinica*.

[24] Pichette V., Leblond F. A. (2003). Drug metabolism in chronic renal failure. *Current Drug Metabolism*.

